RETRACTED

# Changes in Retinal Vessel Flow after Small Incision Lenticule Extraction

**DOI:** 10.1155/2022/8437066

**Published:** 2022-03-09

**Authors:** Qian Tan, Minyi Zhu, Fangfang Du, Xianming Jiang, Xiaoshan Huang, Jingfang Chen, Hongjun Peng, Danyang Wang

**Affiliations:** ^1^Department of Ophthalmology, Shenzhen People's Hospital, Shenzhen 518000, China; ^2^Department of Ophthalmology, The Seventh Affiliated Hospital of Sun Yat-sen University, Shenzhen 518000, China

## Abstract

**Objective:**

In order to analyze changes in retinal vessel flow after small incision lenticule extraction (SMILE).

**Methods:**

A total of 32 patients (62 eyes) who underwent SMILE were enrolled in this prospective study. Optical parameters, including vessel density (VD), and perfusion density (PD) of foveal, parafoveal, and perifoveal regions, respectively, were measured before surgery and at 1 day, 1 week, 1 month, and 3 months postoperation. Preoperative parameters and surgical parameters were recorded.

**Results:**

Significant decreases in VD and PD on postoperative day 1 were detected in all quadrants, both in 3 mm and in 6 mm regions (*P* < 0.001). One month after surgery, VD returned to preoperative levels. None of the preoperative and surgical parameters were significantly correlated with the VD and PD fluctuations (all *P* > 0.05)*. Conclusion*. VD may decrease significantly with regional disparity 1 day after SMILE while recovering at 1 month. Elevation of intraocular pressure due to suction may account for such changes.

## 1. Introduction

Myopia has emerged as a severe public health issue in the last decade and has drawn significant attention to its complex complications worldwide [1]. A meta-analysis predicted that the prevalence of myopia would reach 49.8%, which means that four billion people will suffer from myopia by 2050 [2]. Myopia, especially high myopia, would bring structural changes such as thinning of the choroid and retina, would decrease retinal nerve fiber layer thickness, and may increase the risk of chorioretinal atrophy, lacquer cracks, choroidal neovascularization, and retinal detachment [1, 3]. Changes in retinal and choroidal blood flow are important entry points for studying the histology of myopia progress. Using fluorescein angiography, several reports have demonstrated a reduced blood flow and a decreased retinal vessel diameter in myopic eyes [4, 5]. Optical coherence tomography angiography (OCT-A) was recently developed for retinal vasculature imaging without the use of dye injection. OCT-A allows for quantitative measurements of retinal vessels, including foveal avascular zone (FAZ), vessel density (VD), and perfusion density (PD). VD is quantified by the percentage of the retinal vessel area in the analyzed area. PD is quantified by the total area of perfused vasculature per unit area in a measurement region [6]. Recently, several studies have shown that foveal and perifoveal retinal flow and density decrease with the axial length age, and the degree of myopia increases [7, 8].

RETRACTED

Small incision lenticule extraction (SMILE) is a new pattern of refractive surgery, which marks a paradigm shift in the field of refractive surgery from the conventional flap-based corneal ablative procedures to flap-less extraction [9]. A spate of studies indicated that SMILE surgery has excellent outcomes with good predictability, stability, and effectiveness [10–12]. During SMILE surgery, a curved docking system using a limbal suction mechanism stabilized the cornea. Then, an intrastromal lenticule was created using a femtosecond laser, followed by lenticule separation and extraction by a surgeon. Previous studies have shown that acute elevation of IOP may cause ischemia-reperfusion injury that may induce ganglion cell death and retinal function damage [13–15]. Furthermore, Shoji et al. showed that a change in retinal vessel density could be detected before a change in ganglion cell complex thickness occurs [16]. A sudden spike in IOP was seen in the suction part of SMILE surgery [17]; thus, we hypothesized that retinal flow changes after SMILE would be detected. Since severe retinal ischemia brings about myopia-related retinal complications, specific changes in the degree, duration, and especially the degree of vascular blood flow are worth studying. Seldom studies concentrated on retinal foveal vessel flow change after corneal refractive surgery. Zhang and Chen recently reported that femtosecond laser-assisted LASIK (FS-LASIK) and SMILE surgery could cause a temporary decrease in macular vessel density [18, 19]. However, their follow-up time was limited to only 1 month. The relative longer-term effects of SMILE surgery on retinal vasculature have yet to be investigated, and it remains unclear whether the regions change homogeneously.

This prospective study is aimed at evaluating the changes in retinal vasculature measured by OCT-A and the possible correlated factors of these changes after SMILE surgery.

## 2. Patients and Methods

### 2.1. Patients

The Institutional Review Board of the Seventh Affiliated Hospital of Sun Yat-sen University approved this study. All procedures adhered to the Declaration of Helsinki. Informed consent was obtained from all participants before enrollment. From May to July 2019, 32 patients (62 eyes) undergoing SMILE were enrolled in this prospective study, with 8 males (15 eyes) and 24 females (47 eyes). The inclusion criteria were age 18 years or older, stable manifest refraction within the past two years, corrected distance visual acuity (CDVA) of 20/20 or better, spherical refractive error (SE) of -1.00 to -10.00 diopters (D), and myopic cylinder of -3.00 D. The exclusion criteria were a calculated postoperative residual stromal bed thickness less than 280 *μ*m, abnormal corneal topography, and a past medical history of surgery and systemic conditions that could alter the microvasculature, including diabetes, hypertension, cardiovascular disease, and renal disease. Subjects with clinical symptoms of retinal diseases, glaucoma, neurological diseases, severe dry eye, and corneal diseases were also excluded. Ophthalmologic examinations were performed preoperatively and at 1 day, 1 week, 1 month, and 3 months postoperatively. These examinations included visual acuity (uncorrected distance visual acuity (UDVA)), intraocular pressure (noncontact tonometer (CT.1, Topcon, Japan)), anterior and posterior segment examination (SL.3G, Topcon, Japan), and cycloplegic subjective refraction. Corneal topography, cornea diameter indicated by white-to-white (WTW), and corneal curvature were measured by Pentacam (Oculus, Germany).

RETRACTED

### 2.2. Surgical Techniques

All eyes that underwent SMILE were operated with a VisuMax femtosecond laser system (Carl Zeiss Meditec AG, Jena, Germany) with a 500 kHz repetition rate. Before surgical procedures, proxymetacaine hydrochloride eye drops (Alcaine; Santen Pharmaceutical) were administered as local anesthesia. Laser energy was 110 to 175 nJ. The laser cutting was performed in the sequential four steps: posterior surface of the lenticule (spiral in pattern), lenticule side cut, anterior surface of the lenticule (spiral out pattern), and a cap side cut. The intended thickness of the cap was 110 or 120 *μ*m, and the lenticule diameters were 6.3 to 6.8 mm. A 2 mm incision for lenticule extraction was positioned at 130° with a side cut angle of 90°. After laser scanning was completed, a spatula was inserted through the cut to separate the lenticule. A microforceps was subsequently taken to grasp and remove the lenticule through the small incision. The incision was flushed with a balanced salt solution in the end. All surgeries were performed by the same doctor (WDY). After surgery, eye drops of 0.3% Levofloxacin (Cravit; Santen, Inc., Osaka, Japan) were administered four times daily for 2 weeks. Tobramycin dexamethasone eye drops were used every 2 hours for 1 week, followed by fluorometholone (0.1%) (Flumetholon; Santen, Inc.) four times daily for the following 3 weeks.

### 2.3. OCT-A Data Acquisition and Processing

OCT-A scans were captured with a Cirrus high-definition–OCT prototype AngioPlex instrument using the Optical Micro Angiography algorithm (Carl Zeiss Meditec, Inc., German) under dim circumstances (illumination < 10 lux). The observer who operated the examination was blinded to the study. To avoid the effects of diurnal variations, all measurements were obtained before noon. The refraction was adjusted during examinations until the en face image was clear to eliminate the influence of refraction and magnification. Subjects were asked to remain stable and stare at the center of the cross fixation target, while the effect of eye motion-related artifacts was minimized by tracking eye movements with FastTrac™ retinal-tracking technology. Macular 3 × 3 mm and 6 × 6 mm scans were performed on each patient. Images with a signal intensity over 8 and no distortion and segmentation failure were stored, and scans affected by eye movements or decentration artifacts were discarded and repeated. The software (ver. 10.0) automatically visualized the superficial retinal layer slab (SRL) and deep retinal layer slab. The SRL image was segmented from an inner boundary of the internal limiting membrane (ILM) to the inner plexiform layer (IPL) [20]. The parafoveal region was defined as an annulus with an outer diameter of 3.0 mm and an inner diameter of 1.0 mm. The perifoveal region was described as an annulus with an outer diameter of 6.0 mm and an inner diameter of 3.0 mm. Each of the rings was divided into four quadrants (Figure 1). Parameters analyzed included vessel density (VD) and perfusion density (PD) of the SRL in 3 × 3 mm and 6 × 6 mm scans. Both VD and PD of SRL were calculated in the nasal, temporal, inferior, and superior quadrants of the parafoveal and perifoveal regions. (Figures 1 and 2)

RETRACTED

### 2.4. Statistical Analysis

All statistical analyses were performed using SPSS statistical software for Windows, version 22.0 (SPSS, Chicago, IL, USA). CDVA values were transformed to the logarithm of the minimum angle of resolution (LogMAR) values for statistical analyses. Since most of our data were not normally distributed, generalized estimating equations (GEE) were performed to analyze VD and PD changes in SRL through different time points. ANOVA test compared VD and PD decrease at 1 day postoperatively. Spearman's correlation was used to investigate the associations between SE, AL, Km, WTW, suction time, and OCT-A parameters. A *P* value less than 0.05 was considered statistically significant.

## 3. Results

### 3.1. Demographics

The demographic and clinical information of the subjects is listed in Table 1. LogMAR UDVA showed an improvement from 1.22 (1~1.4) preoperatively to −0.08 (-0.08~-0.08) 3 months after surgery. Postoperative CDVA remained stable among follow-up visits. SE recovered 1 day after surgery and remained stable during the following periods, while the IOP stayed unchanged after 1 week. SMILE procedures were performed uneventfully in all patients without any intraoperative and corneal complications at any postoperative time point.

### 3.2. Vessel Density and Perfusion Density in the Foveal, Parafoveal, and Perifoveal Regions

The vessel density of the foveal, parafoveal, and perifoveal regions significantly changed during the follow-up period (*P* < 0.001, Generalized Estimating Equations). VD of all regions 1 day after surgery was less than those before surgery. At 1 month after surgery, vessel density recovered to preoperative levels and remained stable at 3 months (Table 2). One-way ANOVA reported significant differences in VD and PD among various regions 1 day after surgery, with the parafoveal region showing the greatest reduction, while the perifoveal region showed the least reduction (*F* = 5.029, 19.364, *P* = 0.008, 0.001, ANOVA) (Figure 3).

We further compared vessel density and perfusion density at different locations within the 3 mm and 6 mm region, respectively. Vessel density and perfusion density (varying with quadrants) fluctuated significantly among locations (*P* < 0.001, GEE). Significant decreases in VD between 1 day after surgery and before surgery were detected in all orientations in the 3 mm and 6 mm examinations. PD decreased between 1 day postoperatively and 1 day preoperation in all orientations in 3 mm and 6 mm examinations (Table 3 and 4).

### 3.3. Correlation Analysis

Furthermore, we investigated the parameters that may potentially predict the changes in retinal vessel density of the parafoveal and perifoveal regions 1 day after the surgery. However, neither the preoperative nor surgical parameters mentioned in the methods section were significantly correlated with the changes in retinal vessel density and perfusion densities (*P* > 0.05) (Tables 5 and 6).

## 4. Discussion

Currently, SMILE is safe and effective in treating refractive errors comparable with LASIK [10–12]. Previous studies have shown mild, reversible, and localized macular edema after LASIK in adults [21]. However, previous research rarely focused on the retinal changes after SMILE. Our study indicates that the retinal vessel density and perfusion density may decrease 1 day postoperatively and return to preoperative levels at 1 month, while VD changes vary with quadrants. These findings could provide insight into retinal vessel changes after SMILE.

We found that retinal vessel densities in all directions decreased at 1 day postoperatively compared with the preoperative results (10.65 vs. 8.4), returned to preoperational levels at 1 month, and remained stable at 3 months. This trend is consistent with Zhang et al. and Chen et al.'s research [18, 19], which reported a short-term decrease in macular vessel density after FS-LASIK and SMILE surgery. An experiment showed that, during the application of the suction ring, the axial length increased, and the vitreous base fluctuated [22], which indicated a direct mechanical impact of suction on the retina and subsequent intraocular pressure (IOP) fluctuations. Research on mice suggested that moderate IOP elevation lasting for half an hour decreases retinal blood flow examined with Doppler optical coherence tomography [15]. We then hypothesized that sudden fluctuations in IOP caused by suction and release during the procedure might account for the changes in the retinal vasculature. A study using real-time intraoperative IOP detection found that flap creation with the femtosecond laser increased IOP (81.78 ± 10.55 mmHg) less than flap creation with the microkeratome (122.51 ± 16.95 mmHg) [23], and SMILE surgery could induce a peak IOP of 89.17 ± 22.66 mmHg during suction [17, 23]. It has been reported that when IOP rises above 40 mmHg or when the ocular perfusion pressure decreases below 50 mmHg, autoregulation may be overwhelmed, resulting in optic nerve hypoxia [24]. In addition, every 10 mmHg increase in IOP may lead to a 7.4-8.4% decrease in optic disk blood flow, which may cause retinal ischemia-reperfusion damage [25]. Furthermore, mechanical stretching of the retina during surgery due to suction may also play an important role. Flaxel et al. showed that axial length increases after suction ring application, whereas anterior chamber depth shows no significant difference, suggesting that an anterior forward movement of the vitreous base results in traction on the anterior retina, worsening the ischemia damage [22].

RETRACTED

This article prolonged the observation period to 3 months and found no statistical difference in VD and PD between 1 and 3 months. This was similar to Xu et al.'s results. They measured the choriocapillaris vascular density in LASIK patients and found that the choroid vessel flow decreased on day 1, returned to baseline within 1 month, and remained unchanged over 3 months. The choroidal and retinal changes were considered a stress response to the surgery rather than real injury [26].

We further unprecedentedly reported the disparate changes of retinal vasculature after SMILE between parafoveal and perifoveal regions. Our study showed that both vessel density and perfusion density experienced a more significant reduction in the parafoveal region compared with the perifoveal region. In Chen et al.'s study, the vessel density reduced from 51.77 to 48.45 in the perifoveal area and 52.91 to 48.97 in the parafoveal area 1 day after surgery, with a similar tendency as in our research [18]. Previous studies that focused on retinal thickness after LASIK also found that foveal and parafoveal regions tended to be thicker 1 day after surgery, but not in the perifoveal area [21, 27]. Therefore, we speculate that the use of contact lenses during SMILE may have caused small localized lesions of the macula in the early postoperative period, mainly in foveal and parafoveal retinal regions rather than the perifoveal area. In addition, we also noted a slightly higher decrease in the temporal than the nasal area and a higher reduction in the inferior region than in the superior region. We suspect that the changes in VD and PD that were different among quadrants may be related to the structure and inconsistence distribution of microvasculature in the fovea, which requires further investigation [28].

We analyzed the relationship among vessel density, perfusion density variations and other surgical or demographic parameters. There was no significant relationship between the changes in the retinal vasculature and the axial length, preoperative manifest spherical equivalent, corneal diameter, and suction time. Curiously, suction time was not significantly correlated with the retinal vasculature variation since long-lasting suction time may induce more IOP fluctuations. The expert mode was used in our surgery, and the suction time varied from 29 s to 34 s. We hypothesized that this time variation might not be sufficient to cause significant differences in the retinal vessel fluid between patients. When compared with FS-LASIK surgery, SMILE surgery suction time was much longer (32 s vs. 14 s) [17, 21, 23]. In LASIK surgery, the IOP was elevated only in flap creation procedures, while in SMILE surgery, there was a continuous IOP fluctuation not only in lenticule creation but also in lenticule separation and extraction. Data from Chen et al. and Zhang et al.'s reports also showed that SMILE might induce more VD variations than FS-LASIK, but they used different surgical equipment [18, 19]. Some studies have indicated that a peak IOP higher than 150 mmHg was observed in some femtosecond laser devices, while the peak IOP in VisuMax was significantly lower [29, 30]. This may also be a consideration when comparing SMILE and FS-LASIK and may contribute to the influence of suction on retinal vessel changes.

Although VD and PD decreased postoperatively, CDVA improved significantly after surgery and remained stable during the 3-month follow-up period. The above suggests that retinal vessel density and perfusion density had a limited impact on the visual recovery and safety in SMILE, and reductions in vessel density and perfusion density in all regions are temporary and reversible after surgery.

RETRACTED

There were several limitations in our research. Firstly, we only observed blood vessel changes in myopia patients who underwent SMILE. Due to significant corneal opacity, early postoperative use of corneal bandage contact lens that would lead to inaccurate OCT-A measurements, we did not choose PRK and LASIK patients as the control groups. Secondly, data on deep vessels were not available, as the OCT-A of ZEISS can only provide quantitative data for the superficial retinal capillaries. It is hoped that ZEISS can develop a quantitative analysis of deep vessels as soon as possible. In addition, a larger sample size would be more desirable to achieve a normal distribution in future studies, as parametric statistical tests based on normal distribution could provide higher statistical power and quantitative comparisons.

In summary, our study showed that VD and PD changed over time and varied with quadrants and regions. Suction may be the cause of this. No correlation was found between VD/PD changes and other parameters in the current study. In future studies, comparison with FS-LASIK using the same or different femtosecond laser device may better help reveal the influence of suction time and peak IOP pressure on VD and PD changes.

## Figures and Tables

**Figure 1:** Vessel density (VD) and perfusion density (PD) of different directions. Macular vessel density (a) and perfusion density (b) were separately automatically calculated from ETDRS contours in a 3 mm measuring instrument in five regions (foveal, temporal, superior, nasal, and inferior), respectively. Vascular density (c) and perfusion density (d) were independently measured in three areas: the fovea, the inner ring, and the outer ring in 6 mm detection. (e) and (f) show the abbreviation code of different regions. T1 and T2 refer to the inner and outer area temporal to the macular; N1 and N2 were locations of the regions nasal to macular, respectively; I1 and I2 represent the inner and outer regions inferior to macular, respectively; S1 and S2 refer to the location of the inner and outer rings superior to macular, respectively.

**Figure 2:** VD and PD changes at different time points. (a)–(e) show the retinal vessel density of one person from before surgery to 3 months after surgery. (f)–(j) were the perfusion density of SRL retina presentations from before surgery to 1 day, 1 week, 1 month, and 3 months after surgery.

RETRACTED

**Figure 3:** Fluctuation of PD and VD of different regions in the following periods. VD: vessel density; PD: perfusion density. (a) Macular vessel density in all sections, including the foveal, parafoveal, and perifoveal, decreased around 1 day after surgery and slowly returned to baseline levels within 1 month and remained stable within 3 months. (b) Foveal, parafoveal, and perifovea perfusion density first decreased and then increased to baseline within 1 month.

**Table 1:** Demographic data.

Age (years)	26 (24~28.25)
SE (diopters)	-4.44 (-5.16~-3.23)
AL (mm)	25.05 (24.25~25.82)
UDVA	1.22 (1~1.4)
Km	43.17 (42.37~44.12)
WTW (mm)	11.75 (11.65~11.94)

SE: spherical equivalent; AL: axial length; UDVA: uncorrected visual acuity; Km: mean curvature; WTW: white to white.

**Table 2:** Vessel density and perfusion density before and after SMILE.

	VD of the fovea	VD of the inner ring	VD of the outer ring	PD of fovea	PD of the inner ring	PD of the outer ring
Before surgery	10.65 (8.68~12.85)	22.25 (21.48~23)	18.75 (17.95~19.03)	0.18 (0.14~0.22)	0.39 (0.38~0.4)	0.45 (0.44~0.47)
1 d after surgery	8.4 (6.3~10.43)	19.65 (18.78~21.13)	17.4 (16.3~18.53)	0.14 (0.11~0.18)	0.33 (0.32~0.36)	0.43 (0.4~0.46)
1 w after surgery	9.3 (7.35~12.33)	21.3 (20.13~21.98)	18.4 (17.33~18.8)	0.16 (0.12~0.2)	0.38 (0.36~0.39)	0.45 (0.42~0.47)
1 m after surgery	10.15 (8.23~12.4)	22 (21.2~22.48)	18.7 (18~19.1)	0.17 (0.13~0.21)	0.39 (0.37~0.4)	0.46 (0.45~0.47)
3 m after surgery	9.6 (8.1~11.3)	21.5 (20.7~22.2)	18.5 (17.85~19.1)	0.17 (0.13~0.19)	0.37 (0.35~0.39)	0.46 (0.44~0.47)
Wald chi-square	265.44	30932.20	56440.55	155.60	32812.04	45087.22
*P* value	≤0.001	≤0.001	≤0.001	≤0.001	≤0.001	≤0.001

VD: vessel density; PD: perfusion density.

**Table 3:** Vessel density before and after SMILE.

	Before surgery	1 day after surgery	1 week after surgery	1 month after surgery	3 months after surgery	Wald chi-square	*P*
Fovea	10.65 (8.68~12.85)	8.4 (6.3~10.43)	9.3 (7.35~12.33)	10.15 (8.23~12.4)	9.6 (8.1~11.3)	155.60	≤0.001
S1	22.6 (21.48~23.4)	20.7 (19.18~22.03)	21.8 (20.4~22.58)	22.4 (21.53~23.2)	21.8 (20.6~23)	21399.28	≤0.001
S2	19 (18.2~19.5)	17.85 (16.28~18.9)	18.6 (17.1~19.28)	18.9 (18.3~19.4)	18.6 (18~19.1)	47519.67	≤0.001
I1	22.25 (21.08~23.2)	19.85 (18.4~21)	21 (19.63~22.15)	21.75 (20.73~22.48)	21.3 (20.5~22.5)	10776.32	≤0.001
I2	18.9 (18.2~19.5)	17.7 (16.4~18.63)	18.45 (17.55~19)	18.8 (17.83~19.3)	18.6 (17.95~19.3)	55143.05	≤0.001
N1	22.45 (21.68~23.2)	20.3 (18.68~22.05)	21.55 (20.55~22.48)	22.1 (21.13~22.9)	21.9 (20.9~22.6)	954.15	≤0.001
N2	20.35 (19.78~20.5)	19.95 (18.7~20.3)	20.05 (19.2~20.5)	20.1 (19.75~20.4)	20.1 (19.6~20.4)	65632.76	≤0.001
T1	22.4 (21.1~22.93)	19.6 (17.9~21.1)	20.95 (19.58~21.98)	21.55 (20.7~22.28)	21.3 (20.4~22.1)	865.51	≤0.001
T2	17.55 (16.8~18.43)	15.85 (12.85~16.93)	16.9 (15.25~17.58)	17.25 (15.7~18)	17.1 (16.1~18.05)	2010.06	≤0.001

RETRACTED

**Table 4:** Perfusion density before and after SMILE.

	Before surgery	1 day after surgery	1 week after surgery	1 month after surgery	3 months after surgery	Wald chi-square	*P*
Fovea	0.18 (0.14~0.22)	0.14 (0.11~0.18)	0.16 (0.12~0.2)	0.17 (0.13~0.21)	0.17 (0.13~0.19)	265.44	≤0.001
S1	0.41 (0.39~0.42)	0.37 (0.35~0.39)	0.39 (0.37~0.4)	0.4 (0.39~0.41)	0.39 (0.36~0.41)	26099.71	≤0.001
S2	0.48 (0.46~0.49)	0.45 (0.41~0.48)	0.47 (0.43~0.48)	0.47 (0.46~0.49)	0.47 (0.44~0.48)	38724.68	≤0.001
I1	0.4 (0.37~0.41)	0.35 (0.32~0.38)	0.38 (0.35~0.39)	0.39 (0.37~0.4)	0.38 (0.36~0.4)	15808.35	≤0.001
I2	0.47 (0.45~0.48)	0.44 (0.4~0.46)	0.46 (0.43~0.48)	0.47 (0.44~0.48)	0.47 (0.45~0.48)	42684.55	≤0.001
N1	0.39 (0.38~0.41)	0.36 (0.33~0.39)	0.38 (0.36~0.4)	0.39 (0.37~0.41)	0.39 (0.37~0.4)	11684.74	≤0.001
N2	0.5 (0.49~0.51)	0.49 (0.45~0.5)	0.49 (0.48~0.5)	0.49 (0.48~0.5)	0.49 (0.48~0.5)	1.695	0.193
T1	0.4 (0.38~0.41)	0.35 (0.32~0.38)	0.38 (0.35~0.39)	0.38 (0.36~0.4)	0.38 (0.36~0.4)	16065.95	≤0.001
T2	0.43 (0.41~0.45)	0.38 (0.3~0.42)	0.41 (0.37~0.43)	0.43 (0.38~0.44)	0.42 (0.39~0.44)	12949.67	≤0.001

**Table 5:** Correlations between vessel density differences and preoperational and surgical parameters.

		S1	I1	T1	N1	S2	I2	T2	N2	Fovea	Parafovea	Perifovea
Km	*R*	0.178	0.159	0.138	0.091	0.172	0.119	0.145	0.088	0.201	0.095	0.146
	*P*	0.180	0.233	0.301	0.499	0.197	0.374	0.279	0.510	0.131	0.477	0.274
AL	*R*	-0.080	0.058	-0.038	0.045	0.026	0.036	-0.004	0.041	-0.125	0.018	0.061
	*P*	0.551	0.663	0.776	0.739	0.845	0.787	0.975	0.759	0.351	0.896	0.648
WTW	*R*	-0.059	-0.047	-0.068	-0.194	0.193	0.145	-0.008	0.163	-0.167	-0.152	0.177
	*P*	0.659	0.727	0.614	0.144	0.146	0.279	0.951	0.221	0.209	0.256	0.185
Suction time	*R*	0.056	0.008	-0.052	-0.034	0.255	0.012	0.227	0.007	-0.029	0.042	0.175
	*P*	0.693	0.957	0.716	0.808	0.068	0.930	0.106	0.960	0.838	0.767	0.214
Lenticule diameter	*R*	-0.073	0.030	-0.206	0.073	0.093	0.019	-0.055	-0.070	-0.043	-0.033	-0.043
	*P*	0.608	0.832	0.142	0.607	0.513	0.895	0.699	0.622	0.763	0.817	0.763
SE	*R*	0.021	-0.127	-0.030	-0.097	-0.161	-0.051	-0.234	-0.023	0.008	-0.090	-0.177
	*P*	0.875	0.343	0.824	0.467	0.227	0.706	0.077	0.864	0.951	0.502	0.183
K1	*R*	0.193	0.216	0.132	0.149	0.116	0.082	0.076	0.039	0.234	0.144	0.080
	*P*	0.147	0.103	0.325	0.263	0.388	0.542	0.573	0.770	0.077	0.280	0.549
K2	*R*	0.153	0.078	0.167	0.030	0.194	0.089	0.234	0.114	0.168	0.041	0.193
	*P*	0.252	0.559	0.210	0.823	0.145	0.505	0.077	0.393	0.208	0.761	0.147

Km: mean curvature; K1: flattened curvature; K2: deep curvature; AL: axial length; SE: spherical refractive error; WTW: diameter of cornea indicated by white-to-white.

RETRACTED

**Table 6:** Correlations between perfusion density differences and preoperational and surgical parameters.

		S1	I1	T1	N1	S2	I2	T2	N2	Fovea	Parafovea	Perifovea
Km	*R*	0.252	0.113	0.166	0.019	0.143	0.087	0.137	0.129	-0.034	0.052	0.083
	*P*	0.056	0.399	0.214	0.885	0.284	0.517	0.304	0.334	0.801	0.697	0.538
AL	*R*	-0.174	0.061	-0.022	-0.008	-0.008	0.057	0.022	-0.047	0.137	0.033	0.120
	*P*	0.192	0.648	0.868	0.954	0.954	0.671	0.867	0.729	0.305	0.807	0.371
WTW	*R*	-0.001	-0.058	-0.063	-0.110	0.148	0.132	-0.050	0.241	0.073	-0.143	0.201
	*P*	0.992	0.665	0.638	0.411	0.268	0.325	0.707	0.068	0.587	0.283	0.130
Suction time	*R*	0.015	0.019	-0.033	-0.079	0.242	0.009	0.248	-0.013	0.095	0.103	0.123
	*P*	0.913	0.896	0.815	0.577	0.084	0.951	0.076	0.928	0.503	0.468	0.386
Lenticule diameter	*R*	-0.050	0.027	-0.206	0.165	0.093	0.047	-0.090	-0.046	-0.052	0.044	-0.069
	*P*	0.726	0.851	0.142	0.242	0.513	0.741	0.524	0.746	0.714	0.755	0.625
SE	*R*	0.140	-0.139	-0.053	-0.019	-0.120	-0.028	-0.216	0.147	-0.254	-0.121	-0.120
	*P*	0.296	0.296	0.694	0.886	0.370	0.833	0.103	0.272	0.054	0.365	0.372
K1	*R*	0.259	0.155	0.137	0.067	0.083	0.051	0.059	0.094	-0.037	0.096	0.024
	*P*	0.050	0.246	0.304	0.617	0.536	0.702	0.658	0.483	0.781	0.474	0.857
K2	*R*	0.218	0.045	0.213	-0.036	0.167	0.053	0.238	0.145	-0.006	0.003	0.106
	*P*	0.101	0.735	0.108	0.787	0.211	0.694	0.072	0.279	0.962	0.983	0.431

## Data Availability

The data used to support the findings of this study are available from the corresponding author upon request.
